The article "An Unusual Case of Opacified Intraocular Lens Exchange After 50 Months: A Case Report" was published in 2021. Journal: Cureus.

# An Unusual Case of Opacified Intraocular Lens Exchange After 50 Months: A Case Report

**DOI:** 10.7759/cureus.20193

**Published:** 2021-12-06

**Authors:** Ayesha Ahmed, Bilal Malik, Muhammad Khan

**Affiliations:** 1 Ophthalmology, Aga Khan Health Service, Karachi, PAK; 2 Ophthalmology, Prince Sultan Military Medical City, Riyadh, PAK

**Keywords:** intraocular implants, crystalline lens, opacification, long term complication, viscodissection

## Abstract

A 65-year-old male presented with decreased vision (20/200) from the past nine months after having undergone cataract surgery (phacoemulsification) four years ago. Anterior segment examination revealed diffusely opacified intraocular lens, and he was diagnosed as a case of delayed intraocular lens (IOL) opacification. IOL lens exchange surgery was planned. A per-operative assessment revealed significant fibrosis of IOL with the capsule. Viscoelastic was used for viscodissection, and the IOL was mobilized and removed. Capsular integrity was ensured and achieved, and a new foldable IOL was implanted in the bag. Best-corrected visual acuity (BCVA) after the surgery improved to 20/20. Here, we discuss different IOL exchange techniques and report our successful viscodissection despite significant fibrosis and the time interval of four years since the initial implant.

## Introduction

The leading cause of preventable blindness worldwide is cataracts, accounting for 43.6% of cases in East Asia alone [1]. Cataracts are commonly caused due to aging and are treated with phacoemulsification surgery followed by implantation of an intraocular lens (IOL). Foldable IOLs have commonly been used over the recent decades, and they are made up of various inert materials such as silicone, acrylic, or hydrogel [1]. Occasionally, IOL explantation, either followed by a new IOL implant or without it, may be deemed necessary due to various complications such as incorrect IOL power, dislocation of the IOL, persistent glare, uveitis symptoms, or rarely due to IOL opacification [2]. The reason behind this is unknown; however, studies indicate that the deposition of calcium phosphate hydroxide under the lens surface may be a contributory factor. These deposits have been found to be present in a granular fashion in both the haptics and the optics regions of the lens [3]. As these deposits and consequently the opacification caused by them lead to a substantial decrease in visual acuity, it becomes imperative to perform an IOL exchange using a surgical technique that presents minimal risks [4]. As IOL exchange is a fairly risky surgical procedure that can result in a number of complications, including posterior capsule rupture and zonular dehiscence, predominantly caused by adhesions between the opacified IOL and the capsule [5], we aim to report an interesting case to familiarize ophthalmologists and healthcare professionals with the surgical technique that comes with minimal risks of capsule rupture and zonular dehiscence that we employed to do a successful in-the-bag to in-the-bag IOL exchange after almost four years.

## Case presentation

A sixty-five-year-old man presented with progressively decreasing vision in his left eye for the past nine months. The patient did not give any history of flashes, watering, redness, photophobia, glare, diplopia, or any systemic illness. He, however, gave a history of cataract surgery (phacoemulsification) with a foldable intraocular lens implant in the same eye almost four years (50 months) ago. The surgery was uneventful and had a good visual outcome.

On examination, visual acuity in the right eye was 20/20, while in the left eye, it was 20/200. Pupillary reactions were normal. Anterior segment examination revealed a nondisplaced, diffusely opacified intraocular lens (Figure 1) with a clear cornea and a deep and quiet anterior chamber. The IOL was diffusely opacified, including the double loop haptics, and positioned within the capsular bag. The posterior segment examination was unremarkable in both eyes, and intraocular pressure was 12mmHg and 14mmHg in the right and left eye, respectively.

**Figure 1:** One opacified haptic out of the capsular bag

A diagnosis of delayed opacification of IOL was established, and lens removal and replacement were planned. New K readings were taken, biometry was done, and IOL power was calculated using optical biometry (Zeiss IOLMaster700, ZEISS Medical Technology, Oberkochen, Germany). A foldable, hydrophilic acrylic IOL (Rayner R100, Rayner Intraocular Lenses Limited, West Sussex, United Kingdom) was planned to be implanted in the bag; however, a three-piece IOL for implantation in the ciliary sulcus and an anterior chamber (AC) IOL for implantation in AC was also arranged in order to deal with posterior capsular rupture during the explantation.

Local peribulbar anesthesia was given, and two side-ports were made using a 2.75 mm keratome. The anterior chamber was filled with viscoelastic. Moderate fibrosis of the IOL within the capsular bag was noted; however, viscoelastic was used for viscodissection, and the IOL was mobilized gently within the bag. After the IOL was completely separated from the capsular bag, it was displaced in the AC first, given a nick with scissors near the center of the optic to make it adjustable, and then removed from the side port after enlarging the wound with the keratome (Figure 1 and 2). The integrity of the capsular bag was confirmed (Figure 3), and the new foldable IOL was implanted inside the bag. The patient was advised routine topical postoperative medications, moxifloxacin, dexamethasone, and nepafenac, and called for a follow-up after one and four weeks. Postoperatively the uncorrected visual acuity was 20/40 while best-corrected vision was 20/20, and the new IOL was well centered in the bag.

**Figure 2:** Intact, opacified IOL outside the eye. Notice the small knick on the optic

**Figure 3:** Aphakic, just before inserting the new IOL. Notice the fibrosed yet intact capsule

## Discussion

IOL exchange is an uncommon and challenging procedure, and IOL exchange due to IOL opacification is even rarer, with an incidence of 1% [4]. The cause of opacification is yet unknown, but as mentioned previously, calcium phosphate hydroxide deposits are commonly formed as a result of a chemical reaction and seen under the surface of IOL [3]. However, other researchers reported that the gravitation of calcium ions on hydrogel IOLs was secondary to the migration of silicone from the packaging. The time interval between initial cataract surgery and IOL exchange in our patient was 50 months. This is in comparison to the cases presented by Anil Kubaloglu et al. with 27.69 ± 11.18 months and Seung Mo Kim et al. with 60.4 ± 7.4 months [4,6]. No conclusive pattern could be deduced on the timeline of the opacification.

IOL exchange has many effective surgical techniques [7,8]. Some experimental researchers have tried neodymium-doped yttrium aluminum garnet (Nd: YAG) laser treatment for IOL opacification but were unable to remove the deposits or improve vision. The majority of surgical techniques include removing the IOL after cutting the optic; however, the intraocular scissors may damage the posterior capsule. Posterior capsule rupture has been reported at 12%, 9%, and 8.6% by Kubaloglu, Dagres, and Lee and in their studies, respectively [4,5,9]. Another common complication is zonular dehiscence due to difficulty in separating the haptics from the fibrosed capsule [5]. This is managed by trans-scleral fixation, AC-IOL implant, or removal of prolapsed vitreous, making it very important to have a backup of different lens types [9]. Prolapsed vitreous has a separate incidence of 23% and requires an anterior vitrectomy for its management. Interestingly, the incidence of prolapsed vitreous is very high in patients who had Nd: YAG laser capsulotomy performed on them [10]. 

## Conclusions

The salient feature in our case was the employment of the surgical technique of viscodissection and relieving the adhesions successfully without damaging the capsular bag, and being able to take out the complete IOL intact. As compared to the surgical techniques used in previous studies, viscodissection has proved to be safest as it prevents the complications of zonular dehiscence, vitreous prolapse, and posterior capsule bag damage. We conclude that viscodissection may still be an effective way to remove adhesions and safely remove IOL with minimum complications even after a period of four years of initial IOL implantation.
